# Evaluation of Students' Online Learning Behavior and Perception of Psychological State Based on Data Mining

This article has been retracted.

**DOI:** 10.1155/2022/9867001

**Published:** 2022-06-29

**Authors:** Meng Zhang, Meihui Jia

**Affiliations:** ^1^Department of Literary Law System, Beijing Haidian District Staff University, Beijing 100083, China; ^2^Logistics College, Beijing Wuzi University, Beijing 101149, China

## Abstract

This paper first analyzes the characteristics of students' OLB and stimulates students' online learning motivation based on the locus of control (LoC) stimulation model. Through data mining technology, this paper puts forward the analysis model of OLB, the sequence mining model of OLB, and the interactive model of OLB. Finally, a psychological state perception model based on OLB analysis is constructed; MAE and MSE are used as indexes to compare the fitting effects of GBRT, AdaBoostRegression, LinearSVR, and LinearRegression algorithms on the model. The results show that the relationship between students' psychological state and OLB is very close. While the model constructed has certain predictive ability for students' psychological state perception of OLB, which has certain practical significance for the regulation of students' learning behavior.

## 1. Introduction

The development of Internet technology is constantly adapting to people's needs, and its wide application in the field of education has greatly changed the traditional educational methods, skills, and ideas, and developed rapidly in various forms [1, 2]. How to use the distance education platform for efficient learning has also begun to be concerned by more and more scholars [3]. E-learning usually refers to a process of learning knowledge by means of the network and in an independent or assisted way. Therefore, the analysis of OLB is of great significance to the formulation and development of distance education platform with better learning experience and the more efficient evaluation and accurate guidance of online learning.

Data mining is conducive to the correct choice of decision making. Through statistical analysis of data, useful regular information can be extracted, which plays an important role in avoiding transaction risks for users [4]. In the aspect of education, we can extract certain rules and valuable conclusions from massive learning behavior data through data mining that is used to improve the quality of online teaching and make learning plans, which plays an important role in curriculum formulation, teaching guidance, and learning content [3, 5]. With massive open online courses (MOOCs) becoming a new way for educational materials to reach the public, the research on the mining of MOOC data can help us understand the cultural popularization of different countries and can also learn about the differences in user behaviors, the actual needs of the education market, etc. [6]. But so far, online courses cannot attract learners' attention for a long time. Although many researchers now know that the active learning principle is effective for online learners, the current MOOC teaching methods often allow participants to learn passively, which leads to the unsatisfactory behavior of many online learning participants today [7, 8]. When students are faced with learning tasks, they cannot get a sense of satisfaction and accomplishment. At the same time, learning efficiency is closely related to psychological anxiety and autonomy. Therefore, psychological intervention on students' online behavior can reduce the perceived load and anxiety and improve their learning autonomy.

Therefore, this paper uses data mining technology to analyze learning behavior and then constructs a hierarchical analysis model of learning behavior. Combined with the related research results of online learning in psychology, it finds out the reasons that affect students' learning efficiency and interest points, and gives some psychological suggestions to participants who learn online.

## 2. OLB Based on Psychological Intervention

### 2.1. Characteristics of OLB

Compared with the traditional teaching method in which students passively accept the teacher's knowledge explanation, the learning style, learning interest, and learning autonomy of learners in online learning have changed, and these changes are mainly reflected in the characteristics shown in Figure 1 [9, 10].

#### 2.1.1. Diversified Access of the Network Learning Resource

Traditional learning has to face the shortcomings of face-to-face teaching in class, while online learning has changed the previous teaching mode in a specific classroom with the help of advanced multimedia technology and Internet technology, which can make learners have diversified learning environment and richer access to learning resources.

#### 2.1.2. Diversification and Virtualization of Online Learning Situations

Under the traditional face-to-face teaching environment, teaching and learning generally take place in a fixed and relatively closed environment. Due to various conditions, the teaching mode and teaching environment are characterized by simplification. The innovation of network technology makes online learning have more diverse learning situations where learners can get richer learning experience by using the virtual situation, and gain knowledge and experience.

#### 2.1.3. Autonomy and Individuality of OLB

The development of distance education provides learners with a relatively open lifelong learning system where learners can independently determine learning tasks and learning methods and evaluate learning results according to their own time, environment, and other factors, which makes them have high autonomy and more choices that the learning needs in most environments can be met. When encountering doubts that they cannot answer or have relevant learning experiences, learners can ask for answers and share experiences through posting bars and Weibo, which promotes the communication between online learners and improves the freedom of the information sharing.

### 2.2. Motivation of Students' Online Learning

Learners' different purposes of online learning show different learners' interest in online learning and their desire for knowledge acquisition [11]. Because online learning mainly depends on learners' self-consciousness and self-control, learners may be more or less influenced by some factors in the learning process, including learners' own psychological factors and environmental factors. Moreover, in the face of the huge variety of learning resources in distance education, learners' learning activities may become complicated due to their difficult choices, which has hit the initiative of online learners' autonomous learning, led to some learners' negative neglect in learning, and reduced the learning progress and learning effect. Therefore, it needs to require rational construction of learning resources and personalized recommendation of learning content, so that students can be more active and enthusiastic in learning. The learner's motivation model is shown in Figure 2.

### 2.3. Psychological Intervention Stimulates OLB

Because online learning is not limited by objective environments such as geographical space and time, teachers often cannot communicate with learners offline. In order to improve learners' autonomy and weak control, the model proposes to manage learners' online learning motivation from the perspective of teachers. Combined with the related literature, positive emotion, achievement motivation, and attribution training were used to reduce LoC, which made the experimental subjects more internally controlled. These stimulating strategies were integrated into the online learning process, and a preliminary model of LoC stimulating online learning motivation was constructed. As shown in Figure 3, according to the order of learning, it can be divided into three stages, namely, learning preparation stage, learning development stage, and learning evaluation stage, and positive emotions, attribution training and achievement motivation are the three elements that make the locus of psychological control internalized.

#### 2.3.1. Learning Preparation Stage

There is a negative correlation between positive emotion and LoC and mobilizing college students' positive emotion can make their LoC internally controlled. Therefore, in the learning preparation stage, teachers use the functions of the course learning platform to design a friendly online learning environment. The course syllabus and teaching objectives arouse learners' positive emotions, which make their LoC tend to be internal control. At this stage, students' curiosity, concern, enthusiasm, relaxation, confidence, and other positive emotions can be mobilized by defining appropriate teaching objectives, various preclass teaching materials, and friendly platform interface design so that learners' interest in courses can be improved and their LoC can be controlled. Learners' learning behavior is guided by internal factors, rather than external factors that lead to forced online learning, thus improving motivation of online learning.

#### 2.3.2. Learning Development Stage

In the development stage, there will be a lot of interaction between teachers and learners. Learners can participate in learning activities by reading teaching resources, participating in online discussions, completing course assignments, etc. Teachers can take advantage of the online platform to provide learners with a variety of teaching materials, student-centered teaching strategies and process evaluation that can implement feedback, so as to help learners participate in learning deeply, complete learning tasks better, and achieve teaching results. While completing the learning task, learners will be responsible for their own behaviors according to the task results and teacher feedback. They may think that good feedback is caused by external factors such as good luck, or that bad feedback is caused by external factors such as difficult tasks. This kind of negative attribution will lead students to externalize their LoC, thereby affecting the online learning motivation of college students. Teachers can combine learners' characteristics and their feedback to carry out appropriate attribution training and educational intervention for students with negative attribution.

#### 2.3.3. Learning Evaluation Stage

The evaluation of online learning should not only consist of exam grades and homework evaluation. In order to improve college students' learning motivation and reduce the score of LoC, the evaluation of learners should not simply adopt scores or grades. They should be reasonably praised and criticized in combination with their feedback to teachers during online course learning.

## 3. Analysis Model of OLB Based on Data Mining

### 3.1. Process of Data Mining

Data mining is actually a process of extracting valuable information data or obtaining regular knowledge from massive data [12], which includes four stages, such as data acquisition, data preparation, data mining, and expression of mining results, as shown in Figure 4.

#### 3.1.1. Data Acquisition

Before data mining starts, we must first determine the problem. In this process, data miners need to communicate with users, understand the purpose of data mining, determine the data to be operated and be familiar with the business process of these data.

#### 3.1.2. Data Preparation

It mainly includes three stages: data integration, data selection, and data preprocessing, thus providing the basis for subsequent data processing. Through these operations, noise elimination, repetition elimination, and type conversion can greatly improve the accuracy of subsequent data mining results. Therefore, this stage is to sort out the data to improve the mining quality.

Data integration means that data generated by different data sources are converted and integrated in a specific form.

Data selection represents that after data integration and other processing of the data retrieved in the database, not all the data information obtained is effective for data mining, so it is necessary to select as many relevant data with practical significance as possible.

Data preprocessing includes data denoising and conversion of data type so that these data can be more efficiently applied to data mining systems where the data are preprocessed mainly through data conversion, integration, cleaning, and specification.

#### 3.1.3. Data Mining

After analyzing the user's needs and determining the goal of data mining, an appropriate and efficient method is selected to mine and analyze the data according to the relevant requirements.

#### 3.1.4. Expression of Mining Results

The algorithm of data mining, related technologies, and the quality of preprocessed data may have a certain impact on the results of data mining. If the wrong methods or inappropriate data are adopted, the results of data mining will deviate from people's expectations. Therefore, it is necessary to evaluate the final results and delete irrelevant or redundant results.

### 3.2. Interaction Model of OLB

Under the traditional online teaching mode, teachers and students are separated in time and space, and there is little interaction between learners and teachers. In order to make teachers know students better, we build an OLB interaction model based on learning behavior mining analysis, as shown in Figure 5.

Among them, learners can learn courses, answer questions, and take online tests on the platform. They can also participate in learning forums, interest groups, and other learning activities. While teachers can organize, create teaching resources, and can also guide students according to some learners' learning characteristics. Through the interaction model, managers can have a clear understanding of students' learning behavior.

### 3.3. Analysis Model of OLB

Among the existing learning behavior analysis models, the analysis process of learning behavior is less, and the structure of analysis model of OLB is relatively simple. In this paper, a hierarchical OLB analysis model, which includes data storage, learning behavior mining, and personalized learning, is established on the basis of combining the influencing factors of learning behavior effect, external performance of learning behavior, and analysis strategies of learning behavior, as shown in Figure 6.

The above model is divided into three layers, namely, data storage layer, learning behavior mining analysis layer, and personalized learning layer from bottom to top [13].

1. Data storage layer: data sets provide the underlying support and data support services for the learning behavior analysis model. The data in the data sets come from multiple sources, which are generally log data generated by learners' learning behaviors and behavior data dynamically generated in the learning process.
2. Learning behavior mining analysis layer: it is mainly used to mine and analyze the data from the data set after preprocessing, and to express the learners' characteristics and learning patterns.
3. Personalized learning layer: the results of learning behavior mining are presented to learners and teachers in a visual way so that learners can obtain learning resources that meet their own needs, while teachers can give guidance to learners' OLB according to their learning characteristics, or make appropriate adjustments to teaching content based on this.

### 3.4. Sequence Mining Model of OLB

The purpose of learning sequence mining is to mine and analyze the learning sequences commonly used by learners and obtain valuable learning sequences for adaptive recommendation of learning content. The specific model is shown in Figure 7.

There will be a lot of learning sequences generated by the system, and some effective sequences with high support can be put into the learner strategy library. When the students visit the distance education learning platform, they can match their learning patterns and recommend related learning content.

## 4. Psychological State Perception Model Based on OLB Analysis

### 4.1. Data Preparation

The data source of this experiment is the OLB data of 2020 freshmen in a university, and all the data have been desensitized. In the process of experiment, the data labels are obtained from the depression dimension scores. When regression prediction is made, the depression score is the data label, which constructs the label vector of regression model. When two-class prediction is carried out, according to the results of the national norm, those with depression score greater than 26 are considered to have depression symptoms, whose label is 1. If the depression score is less than or equal to 26, it is considered that there is no depression symptom, and the label is 0. When making multiclassification prediction, the depression scores in [0,26], (26,39], and (39,+∞) are mapped to 0, 1, and 2, respectively, so as to constructs label vector of multiclassification model.

In order to avoid model overfitting and the dependence of model results on data set division, this paper adopts the method of cross-validation to divide the data set into *K* subsets, where *K* − 1 subset is taken as the training set Train and the remaining subset is taken as the Test set. After repeat *K* times, the final result is obtained by averaging the evaluation index of each experiment. In this paper, *K* = 10.

### 4.2. Model Construction

The purpose of constructing the psychological state perception model is to construct an algorithm model with the ability to classify or predict psychological state. The process of constructing the model is to process the original data into two feature vectors *S* and *D*, and each row represents a student's static feature vector and dynamic feature vector respectively, and then associate it with the specific experimental label data. Then, data mining classification or regression algorithm is selected, and the final prediction model is obtained through algorithm training. The specific algorithm process is Algorithm 1.

### 4.3. Evaluation Indicators

For regression problems, mean square error (MSE) and mean absolute error (MAE) are commonly used to measure the difference between the predicted results of the model and the actual results. MSE is calculated as equation (1):

(1) $$\begin{array}{c} \text{MSE}=\frac{1}{N}\sum_{i=1}^{N}{\left(y_{i}-{\hat{y}}_{i}\right)}^{2}. \end{array}$$

While MAE is calculated as equation (2):

(2) $$\begin{array}{c} \text{MAE}=\frac{1}{N}\sum_{i=1}^{N}\left|y_{i}-{\hat{y}}_{i}\right|, \end{array}$$

where *y*_*i*_ indicates the real result, ${\hat{y}}_{i}$ indicates the fitting result, and *N* is the number of samples.

### 4.4. Analysis of Results

Through the regression model, the specific scores of students' psychological depression can be predicted, and the degree of students' psychological depression can be distinguished from a more detailed granularity. The feature matrix is connected with the depression score label, the data set is divided according to cross-validation, and regression prediction is implemented by regression algorithms (e GBRT, AdabooStress, LinearSVR, and LinearRegression). The results are shown in Table 1.

When MSE is used as the index, there is a big gap among the models, and the best algorithm result is 4.07 of LinearRegression; while when the MAE is adopted, the difference between the models is small, and the best result is 1.33 of GBRT. As can be seen from the experimental results that the deviation between the predicted results and the actual results of the model is within an acceptable range, which indicates that the model has certain predictive ability for students' psychological state perception of OLB.

In addition, by aggregating the importance of the feature vectors constructed above, they are divided into static features, learning resource features, learning behavior features, and learning interaction features. The results of feature importance degree of each model are shown in Table 2.

It can be seen from Table 2 that the characteristics of learning behavior account for the highest proportion of importance in each model, with the highest value 0.73, followed by the characteristics of learning interaction, with the highest value 0.60, which shows that there is a close relationship between students' psychological state and OLB.

## 5. Conclusion

In this paper, data mining technology is used to analyze learning behavior, and then a hierarchical learning behavior analysis model is constructed. Combined with the related research results of online learning in psychology, a psychological state perception model based on OLB analysis is constructed. The results show that when the MAE is used as the evaluation index, the errors among the models are small, and the best result is 1.33 of GBRT, which shows that the model has certain predictive ability for students' psychological state perception of OLB. In addition, under different data mining models, learning behavior features account for the highest proportion of importance, with the highest value 0.73, followed by learning interaction features, with the highest value 0.60, which shows that there is a close relationship between students' psychological state and OLB.

## Figures and Tables

**Figure 1:** Characteristics of OLB.

**Figure 2:** Online learning motivation model.

**Figure 3:** Online learning motivation model based on LoC.

**Figure 4:** Data mining process.

**Figure 5:** Interaction model of OLB.

**Figure 6:** Analysis model of OLB.

**Figure 7:** Sequence mining model of OLB.

**Algorithm 1:** Prediction of psychological state perception.

**Table 1:** Comparison of psychological state perception models based on different regression models.

	MAE	MSE
GBRT	1.33	4.89
AdaBoost	1.72	7.31
LinearSVR	1.60	5.22
LinearRegression	1.58	4.07

**Table 2:** Importance analysis of different features.

	GBRT	AdaBoost	LinearSVR	LinearRegression
Static characteristics	0.09	0.11	0.08	0.09
Learning resource	0.18	0.14	0.30	0.27
Learning behavior	0.62	0.73	0.60	0.56
Learning interaction	0.33	0.60	0.53	0.59

## Data Availability

The dataset can be accessed upon request.
